The article "English Feature Recognition Based on GA-BP Neural Network Algorithm and Data Mining" was retracted in 2023. Reasons: unreliable results or conclusions; concerns about the data; concerns about the results or conclusions; concerns about the peer review.

# English Feature Recognition Based on GA-BP Neural Network Algorithm and Data Mining

**DOI:** 10.1155/2021/1890120

**Published:** 2021-08-30

**Authors:** Dan Wu, Yuanjun Shen

**Affiliations:** ^1^School of English Education, Xi'an International Studies University, Xi'an 710128, Shaanxi Province, China; ^2^University College London, WC1E 6BT, London, UK

## Abstract

With the development of society and the promotion of science and technology, English, as the largest universal language in the world, is used by more and more people. In the life around us, there is information in English all the time. However, because the process of manual recognition of English letters is very labor-intensive and inefficient, the demand for computer recognition of English letters is increasing. This paper studies the influence of the parameters of BP neural network and genetic algorithm on the whole network, including the input, output, and number of hidden layer nodes. Finally, it improves and determines the settings and values of the relevant parameters. On this basis, it shows the rationality of the selected parameters through experiments. The results show that only GA-BP neural network and feature data mining algorithm can complete feature extraction and become the main function of feature classification at the same time. After enough initial data sample analysis training, the GA-BP neural network was found to have good data fault tolerance and feature recognition. The experimental results show that the genetic algorithm can find the best weights and thresholds and the weights and thresholds are given to the BP neural network. After training, the recognition of handwritten letters can be realized. Finally, the convergence of the two algorithms is compared through experiments, which shows that the overall performance of the BP neural network algorithm is improved after genetic algorithm optimization. It can be seen that the genetic algorithm has a good effect in improving the BP neural network and this method has a broad prospect in English feature recognition.

## 1. Introduction

 Neural network is a mathematical model network composed of several simple units on the basis of simulating a biological prototype, which has the characteristics of extensive parallel interconnection [1]. The structure of the platform regulation mechanism is that it can effectively simulate the different interactions and reactions of the real-world biological nervous system to all activities of different organisms in the natural biological world in the real world [2]. The neural network is composed of a “simple unit.” In the biological neural network, neurons, as the most basic components, not only exist in large quantities but also connect with each other. When one of the neurons is activated to produce “excitation,” the “excitation” will be transmitted to another neuron through the transmission of chemical substances and the downstream reaction will be guided by changing the potential of other neurons. When the “threshold” is exceeded, the amplitude of potential changes increases and neurons can conduct this process after activation.

The article "English Feature Recognition Based on GA-BP Neural Network Algorithm and Data Mining" was retracted in 2023. Reasons: unreliable results or conclusions; concerns about the data; concerns about the results or conclusions; concerns about the peer review.

As an algorithm model, the artificial neural network is a kind of neural network based on the known principles of biological neural networks, which is constructed by artificial simulation and realizes specific functions through similar processes [3]. It is a mathematical model of the theoretical basis of human brain neural network and an information processing system based on imitating the biological brain neural network. It not only has the ability of self-organization and self-learning but also has other advantages, such as distributed storage and parallel processing of related information [4]. In recent years, the research in artificial neural network has been paid more and more attention and its system category is also expanding. Generally, the artificial neural network is divided into two types based on its structural characteristics; one is forward network and the other is feedback network. This research adopts the BP network which is a typical forward network.

Backpropagation algorithm (BP) was proposed by Alarifi et al. in the paper published in the international journal *Nature*, which is essentially a multilayer perceptron [5]. The BP neural network has many advantages. Compared with the previous algorithms, it has better classification ability. In the optimization of the new-generation neural network, it also has the ability of multidimensional function mapping. Compared with the simple perceptron, it expands the scope of solving problems, which cannot be solved in many previous studies and have been broken through the limitations of the algorithm [6, 7]. Its structure mainly includes three components: input layer, hidden layer, and output layer. In essence, it takes the square of network error as the objective function and uses the gradient descent method to calculate the minimum value of the objective function [8].

The BP neural network has received significant attention since it came out. With the development of science and technology, it is increasingly widely used to solve a variety of practical problems. As a typical forward neural network, the BP neural network is trained on the basis of error backpropagation algorithm. In the process of training, the data is continuously transmitted through forward propagation and error backward transmission and the weight threshold can be updated in real time through the algorithm. On the one hand, in this process, how to determine the weight and threshold of the first forward propagation process is analyzed, that is, how to initialize the weight and threshold. On the other hand, after selecting the initial parameters, the gradient descent algorithm takes the initial parameters as the starting point to optimize and update the parameters.

The article "English Feature Recognition Based on GA-BP Neural Network Algorithm and Data Mining" was retracted in 2023. Reasons: unreliable results or conclusions; concerns about the data; concerns about the results or conclusions; concerns about the peer review.

With the wide utilization of the BP neural network, many problems are solved by its advantages. At present, there is no clear criterion for the selection of BP neural network structure, which can only be set by people's experience. If there are too many choices of network layers, although the accuracy can be improved to a certain extent, the complex structure may lead to unsatisfactory effects in training and a large deviation will occur once the actual situation is encountered. If the number of network layers is small, although the training time is reduced, it also increases the probability of nonconvergence of the whole neural network. Therefore, the determination of the layer of BP neural network should not only be based on the actual requirements but also ensure the training effect of the network. Genetic algorithm uses its own advantages to combine with some other algorithms, such as neural algorithm, which will play a positive role in promoting the development of intelligent algorithms.

In this study, based on the establishment of the BP neural network, genetic algorithm is introduced for further optimization. At the same time, the genetic algorithm is introduced to improve the advantages of the combined algorithm. This optimization process is divided into three steps: the first is to determine the structure of BP neural network, the second is to optimize the genetic algorithm, and the last is to predict the BP neural network through experiments [9, 10]. The first part is mainly about setting parameters and the design of data input function and output function, so as to determine its basic structure [11]. On the basis of structure determination, genetic algorithm is adjusted to optimize the relevant parameters [12–14]. In the last step of the prediction process, after the genetic algorithm optimization, the initial weight threshold assignment of the original BP neural network is optimized and the optimization process of the neural network algorithm can be completed after the input data is trained [15].

In order to meet further extensive needs of English feature recognition, we will design an English feature recognition system, in which a very important step is to use data mining algorithm to extract and array English alphabet features for classification and recognition optimization [16, 17]. Data mining covers a very wide range and interacts with the contents of multiple disciplines. From the initial simple query of data, it is expanded step by step to the extraction of data, mining the knowledge of specific content and classifying it, which provides quite powerful data support for decision-making in many business models [18, 19]. In today's network computing field, it has become a hot research topic [20].

The article "English Feature Recognition Based on GA-BP Neural Network Algorithm and Data Mining" was retracted in 2023. Reasons: unreliable results or conclusions; concerns about the data; concerns about the results or conclusions; concerns about the peer review.

In the field of pattern recognition, English feature recognition, namely, letter recognition, is a valuable subject with a certain economic effect and wide application scope [21, 22]. For recognition of English letters, there are many specific implementation methods and there are different solutions for different conditions [23, 24]. This study aims to realize English feature recognition based on the BP neural network optimized by genetic algorithm and data mining, and through experimental verification on the optimized neural network, the genetic algorithm is found to have a good effect in improving the BP neural network, and this system has a broad prospect in the research of English feature recognition, which provides a theoretical basis for the establishment of related systems in the future.

## 2. Design of the English Feature Recognition System

In order to study the recognition of English features, we need to carry out the pattern recognition process in this study. The application fields of pattern recognition are very wide, as shown in Figure 1, which is the specific process diagram of pattern recognition.

Before the recognition of letters, we must first preprocess the letters. Here, we use the single-pixel feature extraction method; that is, the image is segmented according to a certain size and proportion to get a certain number of sub-blocks containing different information. We scan and recognize the segmented letter graphics and digitize all the 26 English letters through the 5 x 7 grid as shown in Figure 2. This process is a crucial step in English letter image recognition. After processing, the location with data is set to 1 and other locations are set to 0. Shown in Figure 2 is the digitization process of English letters. For example, if the letter A is digitized, the corresponding vector should be letter *a* = [00100010101010001111000110001].

Through the digital processing of 26 English letters, we get the processed data and complete the process of English feature extraction. Next, we will use the algorithm to classify and summarize the data, which will provide the basis for the construction of the feature recognition system. As can be seen from the process in Figure 2, each English letter can be converted into a 35-element vector by numerical processing. All the 26 English letter digital processing data are organized and summarized into a unified input vector matrix, which is used as the input sample of the BP neural network that we will build next.

The article "English Feature Recognition Based on GA-BP Neural Network Algorithm and Data Mining" was retracted in 2023. Reasons: unreliable results or conclusions; concerns about the data; concerns about the results or conclusions; concerns about the peer review.

## 3. English Feature Recognition System Based on the GA-BP Neural Network

### 3.1. Establishment of the BP Neural Network

The BP neural network is structurally divided into three basic components [25]. As shown in Figure 3, the three components are the input layer for receiving information, the hidden layer for processing information, and finally the output layer for obtaining results [26]. In general, the number of input and output layers is set to 1 by default, and then the number of hidden layers is greater than or equal to 1. After the weights are connected, the three components are connected to form a complete BP neural network. Its basic structure is shown in Figure 3.

We can assume that in the structure of BP neural network, the number of nodes in the input layer, hidden layer and output layer is *n, q*, and *m*, respectively. Let *v*_*ki*_ be the connecting weight between the input layer and the hidden layer. Let the output layer and the hidden layer be connected and the weight of the two be *w*_*jk*_. The output of hidden layer node is as follows:

(1) $$\begin{array}{c} z_{k}=f1\left(\sum_{i=0}^{n}v_{ki}x_{i}\right). \end{array}$$

Here, *f*_1_ represents the transfer function in the hidden layer. Let *f*_2_ be the processing function of the output layer; then, the data is substituted into *f*_2_ to get the final output:

(2) $$\begin{array}{c} y_{j}=f_{2}\left(\sum_{k=0}^{q}w_{jk}z_{k}\right). \end{array}$$

The input learning sample is *P*, represented by *x*^1^, *x*^2^,…, *x*^*p*^. After the sample *P* is transformed into data, it is brought into the BP neural network and we obtain the output to get the value *y*_*j*_^*p*^. Setting up *η* in order to get the desired output, the expected output *t*_*j*_^*p*^ and the actual output *y*_*j*_^*p*^ are substituted into the square error formula, and the error of the *P* − th sample is obtained:

(3) $$\begin{array}{c} E_{p}=\frac{1}{2}\sum_{j=1}^{m}{\left(t_{j}^{p}-y_{j}^{p}\right)}^{2}. \end{array}$$

For *P* samples, the global error is

(4) $$\begin{array}{c} E=\frac{1}{2}\sum_{p=1}^{p}\sum_{j=1}^{m}{\left(t_{j}^{p}-y_{j}^{p}\right)}^{2}\\ =\sum_{p=1}^{p}E_{p}. \end{array}$$

The output layer weights change as follows. The calculated single error is superimposed, and *W*_*jk*_ is adjusted according to the superimposed result, so as to reduce the global error *E* and improve the accuracy:

(5) $$\begin{array}{c} \Delta w_{jk}=\sum_{p=1}^{p}\left(-\eta \frac{\partial E}{\partial w_{jk}}\right), \end{array}$$

where *η* represents the learning rate.

The article "English Feature Recognition Based on GA-BP Neural Network Algorithm and Data Mining" was retracted in 2023. Reasons: unreliable results or conclusions; concerns about the data; concerns about the results or conclusions; concerns about the peer review.

The error signal is defined as

(6) $$\begin{array}{c} \delta_{yj}=-\frac{\partial E}{\partial S_{j}}. \end{array}$$

First of all,

(7) $$\begin{array}{c} \frac{\partial E_{p}}{\partial y_{j}}=-\sum_{k=1}^{m}\left(t_{j}^{p}-y_{j}^{p}\right). \end{array}$$

Furthermore,

(8) $$\begin{array}{c} \frac{\partial y_{j}}{\partial S_{j}}=f_{2}\left(S_{j}\right). \end{array}$$

It is the extreme component of the output layer transfer function. Therefore,

(9) $$\begin{array}{c} \delta_{yj}=\sum_{j=1}^{m}\left(t_{j}^{p}-y_{j}^{p}\right)f_{2}\left(S_{j}\right). \end{array}$$

From the chain theorem,

(10) $$\begin{array}{c} \frac{\partial E_{p}}{\partial w_{jk}}=-\sum_{j=1}^{m}\left(t_{j}^{p}-y_{j}^{p}\right)f_{2}\left(S_{j}\right)z_{k}. \end{array}$$

According to formula (10), in the output layer, the weight changes are as follows:

(11) $$\begin{array}{c} \Delta w_{jk}=\sum_{p=1}^{p}\sum_{j=1}^{m}\eta \left(t_{j}^{p}-y_{j}^{p}\right)f_{2}\left(S_{j}\right)z_{k}. \end{array}$$

The change of hidden layer weight is as follows:

(12) $$\begin{array}{c} \Delta v_{ki}=\sum_{p=1}^{p}\left(-\eta \frac{\partial E_{p}}{\partial v_{ki}}\right). \end{array}$$

The error signal is defined as

(13) $$\begin{array}{c} \delta_{zk}=-\frac{\partial E_{p}}{\partial S_{k}}. \end{array}$$

Among them,

(14) $$\begin{array}{c} -\frac{\partial E_{p}}{\partial z_{k}}=-\sum_{j=1}^{m}\left(t_{j}^{p}-y_{j}^{p}\right)\frac{\partial y_{j}}{\partial z_{k}}. \end{array}$$

The chain-dependent theorem is as follows:

(15) $$\begin{array}{c} \frac{\partial y_{j}}{\partial z_{k}}=f_{2}\left(S_{j}\right)w_{jk},\\ \frac{\partial z_{j}}{\partial S_{k}}=f_{2}\left(S_{j}\right). \end{array}$$

It is the partial differential of the hidden layer transfer function. Therefore,

(16) $$\begin{array}{c} \delta_{zk}=-\frac{\partial E_{p}}{\partial S_{k}}=\sum_{j=1}^{m}\left(t_{j}^{p}-y_{j}^{p}\right)f_{2}\left(S_{j}\right)w_{jk}f_{1}\left(S_{k}\right). \end{array}$$

From the chain theorem, we can get that

(17) $$\begin{array}{c} \frac{\partial E_{p}}{\partial v_{ki}}=-\sum_{j=1}^{m}\left(t_{j}^{p}-y_{j}^{p}\right)f_{2}\left(S_{j}\right)w_{jk}f_{1}\left(S_{k}\right)x_{i}. \end{array}$$

According to formula (17), the change of weight in hidden layer is as follows:

(18) $$\begin{array}{c} \Delta v_{ki}=\sum_{p=1}^{p}\sum_{j=1}^{m}\left(t_{j}^{p}-y_{j}^{p}\right)f_{2}\left(S_{j}\right)w_{jk}f_{1}\left(S_{k}\right)x_{i}. \end{array}$$

With the development of science and technology, the BP neural network has been widely used by many people. For example, the existence of local minimum uses the BP neural network algorithm to solve some complex problems; it will be deadlocked, and the local minimum will lead to the expected results. In the BP neural network, the initial weights will ultimately affect the convergence results. In the above situation, if we fall into the deadlock of the local minimum, the selection of the initial weights will also have errors. If we choose different values, we will get different local minima. In this case, the accuracy of BP neural network cannot be guaranteed.

The article "English Feature Recognition Based on GA-BP Neural Network Algorithm and Data Mining" was retracted in 2023. Reasons: unreliable results or conclusions; concerns about the data; concerns about the results or conclusions; concerns about the peer review.

### 3.2. Using Genetic Algorithm to Optimize the BP Neural Network

In order to make up for some problems that cannot be ignored in the BP neural network, genetic algorithm is introduced to further optimize it. Genetic algorithm is a parallel random search optimization method which is artificially constructed by simulating the relevant theoretical mechanism of biological genetic evolution in nature. Based on the principle of “survival of the fittest,” which is well known in genetics, this process is introduced to further optimize the parameters. Through the calculation of fitness function and according to the three processes of selection, crossover, and mutation in genetic mechanism, the individuals with good fitness value are selected. The basic process is shown in Figure 4.

There are also three basic steps to optimize BP using genetic algorithm. Firstly, the infrastructure of neural network needs to be determined and then the neural network prediction is carried out after optimization. The basic purpose of optimization is to simulate the genetic mechanism of natural organisms, and then, the input data samples are optimized to get better initial weights and threshold values, then converted into new data samples, and then reentered into the BP neural network, finally finding the optimal individuals through the basic steps of genetic algorithm selection, crossover, and variation.

In genetic algorithm, in order to facilitate the calculation of individuals in the algorithm, these feasible solutions need to be coded. It can be seen that chromosome coding is an important problem to be dealt with first in the process of optimization. Among the three different coding methods, we use the binary coding method to transform the coding based on the experimental purpose of this study. In this coding, the basic form is mainly composed of 0 and 1, which is very convenient for operation. At the same time, this coding method is more convenient and easier to carry out cross and mutation operations in the process of genetic algorithm optimization and improve the success rate. At the same time, its shortcomings are also very obvious. When one of the individual coding strings is too short, the experimental results will not reach the expected accuracy. If the coding string is too long, the computation will be improved due to the increase of the number of codes, which leads to the weakening of the performance of the algorithm.

The article "English Feature Recognition Based on GA-BP Neural Network Algorithm and Data Mining" was retracted in 2023. Reasons: unreliable results or conclusions; concerns about the data; concerns about the results or conclusions; concerns about the peer review.

The optimization process of genetic algorithm needs to determine the relevant parameters of GA at the beginning. The important parameters are population size *S*, iteration times, cross probability *P*_*c*_, and mutation rate *P*_*m*_. In the above content, we have determined the parameters of BP neural network and we will not go on too much elaboration in this section. Then, we code individuals and screen populations to a certain extent through a process similar to the evolution of nature. Then, the current individuals are crossed and mutated by the cross probability *P*_*c*_ and the mutation rate *P*_*m*_, and a new population is generated, among which *P*_*i*_ is the most adaptable individual. By repeating the previous several parts, after meeting the conditions, the target group of a generation is finally obtained. We take the individual from the target group and input it back to the network system to continue the next calculation process, so we can get the optimized BP neural network. The specific flow is shown in Figure 5.

In many practical models of BP neural network, it is not difficult to analyze that although BP neural network has many advantages of being fast and bright, there are still some shortcomings that need to be made up, such as the characteristics of random initial weights of the network, which will make the experimental effect not meet the expectations. In this study, genetic algorithm is used to optimize and improve the original BP neural network. In the case of preserving the original advantages of BP neural network, genetic algorithm can search the optimal value in a large range of massive data, which further makes up for the defects in BP neural network. Combining the two algorithms can give full play to the advantages of the two algorithms. The experimental results are better than expected.

## 4. Experimental Parameter Setting and Result Analysis

### 4.1. Experimental Parameter Setting

The application range of data mining is very wide, and its process is mainly through the joint calculation of a variety of algorithms to search the target data information in the complex and large number of data samples. There are many ways of data mining, and it is very important to choose the most suitable one according to the characteristics of different methods. These methods all have a common theoretical basis, that is, to get the desired information from the data samples through algorithm calculation. In our study, the corresponding English features are extracted from the specific images of 26 English letters, and on this basis, the data samples of 26 letters after digital processing are classified to provide the classification basis for the subsequent letter recognition. The specific process is shown in Figure 6.

The article "English Feature Recognition Based on GA-BP Neural Network Algorithm and Data Mining" was retracted in 2023. Reasons: unreliable results or conclusions; concerns about the data; concerns about the results or conclusions; concerns about the peer review.

After digital processing of 26 letters, we then explore the influence of the number of nodes in the BP neural network optimized by genetic algorithm on the final convergence result. If the number of nodes in the hidden layer is relatively small in the network, it will make the learning speed increase and pay a certain price, for example, the network learning ability will be reduced. But, the number of nodes is not the better choice. If we choose too many node number parameters, the convergence ability of the model will increase simultaneously, but there will be some problems such as extremely long training time. Therefore, the optimal value must be selected carefully according to the actual situation in the selection of node number. For the selection of the number of related nodes, the reference formula can be referred as follows:

(19) $$\begin{array}{c} n_{1}=\sqrt{n+m}+a, \end{array}$$

where *n* is the number of neurons in the input layer; *m* is the number of neurons in the output layer; *n*_1_ represents the number of neurons in the hidden layer; and *a* represents a random natural number between 1 and 10. The number of nodes is verified by experiments, and the results are shown in Figure 7.

The results in Figure 7 show that, consistent with our previous theoretical analysis, initially, with the increase of the number of hidden layer nodes, the recognition accuracy also increases, but with the further improvement of the number of nodes, beyond a certain optimal range, although the recognition accuracy improves, the efficiency of the whole network model processing data begins to decline. Therefore, we choose the best number of nodes to seek the balance between the recognition accuracy and the performance of the network model.

### 4.2. Analysis of Experimental Results

In practice, we use experimental prediction analysis and cross validation to determine the accuracy of the network algorithm system. We use this method to calculate and verify the accuracy of the 26 English letters in the data set after digital processing.

Figure 8 shows that the classification accuracy values of different 26 English letter samples are not the same. Among them, the letter A may have the highest classification accuracy because of its unique shape among the 26 letters. On the contrary, the shape of the letter H is closer to other letters, so its eigenvalues are closer to other letters, which increases the probability of its being wrongly identified.

The article "English Feature Recognition Based on GA-BP Neural Network Algorithm and Data Mining" was retracted in 2023. Reasons: unreliable results or conclusions; concerns about the data; concerns about the results or conclusions; concerns about the peer review.

Next, we further compared the performance changes of the optimized and unoptimized BP neural networks, compared and tested the differences of the running time and recognition rate before and after the optimization of the genetic algorithm, and expressed them in the form of charts (Figure 9). The data were statistically analyzed with SPSS18.0, the independent sample *T* test was performed, and *P* < 0.05 meant significant difference.

In the test interface, we first collect the specific running time and recognition accuracy of BP neural network in the calculation process of single letter recognition. Then, we collect the optimized BP neural network to calculate the running time and recognition accuracy of the same data sample. From the results, after the genetic algorithm optimization, both the running time and the recognition accuracy are improved to a certain extent.

From the analysis of the above results, compared with the BP neural network alone, the curve reached the expected error faster after using the optimized BP neural network, which proves that the optimized BP neural network is much better in effect than the unoptimized BP neural network, and it also greatly reduces the training time and improves the cost benefit.

In addition, we also use experiments to further verify the performance difference of BP neural network algorithm before and after genetic algorithm optimization, and the results are shown in Figure 10. Under the test of genetic iteration times, BP iteration times, running time, and recognition accuracy, the BP neural network optimized by genetic algorithm has a very significant advantage. Not only its running time is greatly shortened, but also the recognition accuracy is improved by nearly 2%.

This paper analyzes the BP neural network and genetic algorithm in the setting of each parameter on the influence of the whole network, including input, output, and hidden layer node number, as well as step size and mean square error, and finally determine the value of each parameter, through experiments to confirm the rationality of these parameters. The experimental results show that the genetic algorithm can find the best weights and thresholds, and the weights and thresholds are assigned to the BP neural network, which can realize the recognition of English letters after training. Finally, the convergence condition of the two algorithms is compared by experiments, and the convergence time of the improved algorithm is shorter and the accuracy is higher than that of the traditional BP neural network. It can be seen that genetic algorithm has a good effect on improving BP neural network, and this method has a broad prospect in English character recognition and can be applied to a variety of English-based fields.

The article "English Feature Recognition Based on GA-BP Neural Network Algorithm and Data Mining" was retracted in 2023. Reasons: unreliable results or conclusions; concerns about the data; concerns about the results or conclusions; concerns about the peer review.

Computer image recognition technology has been applied in many fields such as public security, biology, industry, agriculture, transportation, and medical treatment, for example, traffic license plate recognition system. With the continuous development of computer technology, image recognition technology is constantly optimized and its algorithm is constantly improved. Image is the main source of human information acquisition and exchange, so image recognition technology related to the image must be the focus of future research. Since the computer image recognition technology is likely to emerge in more fields, its application prospects are unlimited, and human life will be more inseparable from the image recognition technology.

## 5. Conclusion

This paper uses genetic algorithm to optimize BP neural network, and with the aid of data mining algorithm to classify English alphabet features, the construction of the English feature recognition system is realized. Using genetic algorithm to optimize BP neural network not only makes up for the original defects of the BP neural network but also can give full play to the advantages of the combination of the two algorithms. The results show that the GA-BP neural network constructed in this study has achieved a good level of fault tolerance and recognition accuracy. The construction of this system has formed an effective method for English feature recognition, which has a certain universal value. There are also some deficiencies in the experimental process of this paper. In terms of quantization of English character images, only standard characters are assumed to be recognized, without considering the situation of handwritten characters. In the future, we should consider the various situations of the target and improve the identification method according to the actual situation. The feature extraction can be further optimized, and other feature extraction methods can be considered to improve the stability and accuracy of character features, so as to improve the recognition rate of the system. In conclusion, with the deepening of scientific research, people have increasing demands for English feature recognition. The recognition of English letters will be an important field in the future development of the neural network system. The GA-BP neural network and data mining system constructed by this research provide a theoretical basis for the optimization of the English feature recognition system in the future.

The article "English Feature Recognition Based on GA-BP Neural Network Algorithm and Data Mining" was retracted in 2023. Reasons: unreliable results or conclusions; concerns about the data; concerns about the results or conclusions; concerns about the peer review.

## Figures and Tables

**Figure 1:** Process of the recognition system.

**Figure 2:** Letter digital processing.

**Figure 3:** Structure of the BP neural network.

**Figure 4:** The optimization process of the BP neural network by genetic algorithm.

**Figure 5:** GA-BP neural network.

**Figure 6:** Data mining.

**Figure 7:** The influence of the number of hidden layer nodes on the system.

**Figure 8:** The number of samples and classification accuracy of each of the 26 categories of handwritten letters.

**Figure 9:** System comparison module.

**Figure 10:** The effect of neural network before and after optimization.

## Data Availability

The data used to support the findings of this study are available from the corresponding author upon request.
